# Video Abnormal Event Detection Based on One-Class Neural Network

**DOI:** 10.1155/2021/1955116

**Published:** 2021-09-28

**Authors:** Xiangli Xia, Yang Gao

**Affiliations:** ^1^Chongqing Key Laboratory of Spatial Data Mining and Big Data Integration for Ecology and Environment, Chongqing Finance and Economics College, Chongqing 401320, China; ^2^School of Mechanical and Electrical Engineering, Chengdu University of Technology, Chengdu 610059, China

## Abstract

Video abnormal event detection is a challenging problem in pattern recognition field. Existing methods usually design the two steps of video feature extraction and anomaly detection model establishment independently, which leads to the failure to achieve the optimal result. As a remedy, a method based on one-class neural network (ONN) is designed for video anomaly detection. The proposed method combines the layer-by-layer data representation capabilities of the autoencoder and good classification capabilities of ONN. The features of the hidden layer are constructed for the specific task of anomaly detection, thereby obtaining a hyperplane to separate all normal samples from abnormal ones. Experimental results show that the proposed method achieves 94.9% frame-level AUC and 94.5% frame-level AUC on the PED1 subset and PED2 subset from the USCD dataset, respectively. In addition, it achieves 80 correct event detections on the Subway dataset. The results confirm the wide applicability and good performance of the proposed method in industrial and urban environments.

## 1. Introduction

As the demand for social public safety continues to grow, surveillance cameras have been widely deployed as urban infrastructure to provide data sources for video analysis. However, one of the main challenges faced by surveillance video analysis is the detection of abnormal events. In recent years, this labor-intensive task has been designed as an anomaly detection problem [1–3], which aims to identify unexpected events or patterns. Different from the classification and recognition problems in traditional computer vision, anomaly detection has some specific characteristics. First, it is very difficult to list all possible abnormal samples. Second, because the number of occurrences is very small, it is also very difficult to collect enough abnormal samples. In order to solve these problems, one of the most popular methods is to use videos of normal events as training data to learn the model and then judge the samples that do not conform to the learned model as abnormal events. Based on the summary of previous literatures, the present methods can be mainly divided into three categories. The first ones are the distance-based methods [4, 5]. This type of method starts with training the model based on the training samples and measures the deviation from the model to determine the test sample. The abnormal score of the sample is used to determine the abnormality. In [4], the researchers first used the noise reduction self-encoding to extract the appearance and motion characteristics of video blocks and then trained one-class support vector machine (SVM) to achieve anomaly detection. In [5], the anomaly scores were obtained by merging feature changes extracted from pretrained convolutional neural networks. The second ones are probability-based ones [6, 7]. This type of method is similar to the distance-based method, except that the detection model has a probabilistic interpretation, such as a probability graph model or a high-dimensional probability distribution. In [6], the researchers proposed a hybrid dynamic texture representation event, which modeled the hybrid dynamic texture generation process, and performed anomaly detection based on the discriminant significance hypothesis test. In [7], the multiple fixed position monitors were used to extract the optical flow field and calculated the possibility of observation based on the distribution stored in the monitor buffer. The third ones are reconstruction-based methods. This type of method decomposes the input into several common components and then reconstructs the input through these components, thereby minimizing the reconstruction error. Generally, the samples with large reconstruction errors are judged as abnormal ones. Common reconstruction methods include sparse reconstruction [8], autoencoding reconstruction [9, 10], etc.

In recent years, under a data-driven framework, deep learning technologies such as deep neural networks (DNNs), convolutional neural networks (CNNs), autoencoder (AE), and generative adversarial nets (GANs) [11] have been applied in computer vision, speech recognition, natural language processing [12,13], and other fields, which have achieved excellent performance. In fact, deep learning techniques have also been applied to solve anomaly detection problems, such as documents [4, 7, 10]. They are mainly based on two ideas. The first one is to provide higher-level feature representations in addition to manual features. It is based on the idea of CNN, which performs high-level feature representation on video frames through a pretrained network on image classification tasks [8, 14]. Another idea is to use AE [10] or GAN [15] to learn to reconstruct or predict normal video frames and then use the reconstruction error to determine the anomalies [16–21]. Different from the above methods, this paper proposes a new distance-based anomaly detection method. This method is based on one-class neural network (ONN), which is an extension of one-class classifiers under the framework of deep learning. Different from other distance-based anomaly methods, the data representation in the hidden layer is directly driven by ONN, so it can be designed for anomaly detection tasks. In other methods, manual features or features extracted by CNN are often used. It is completely independent and cannot be jointly optimized. ONN combines the layer-by-layer data representation capability of the autoencoder and the one-class classification capability to obtain a hyperplane, which separates all normal samples from abnormal ones. The proposed method trains ONN to detect the appearance anomaly and motion anomaly by separately training the local area blocks with the same size of the video frame and the optical flow map. Then, it merges the two to determine the final detection result. The experimental results on two public datasets show that the detection performance of the proposed method outperforms some state-of-the-art ones.

## 2. Principle of the Algorithm

The overall process of the method proposed in this paper is shown in Figure 1. In the training phase, the RGB images and optical flow diagrams of the training samples are intensively sampled. Then, two AE networks are learned separately, and the encoder layer of the pretrained AE and the ONN is copied to jointly optimize the parameters and learn the anomaly detection model. In the test stage, the RGB map and optical flow map of a given test area are input into the appearance anomaly detection model and the motion anomaly detection model. The two output scores are fused to set the detection threshold to determine whether the area is abnormal. In this section, we first briefly explain the autoencoder and a type of support vector machine. Afterwards, we introduce the principle of the ONN model and the process of the video abnormal event detection algorithm based on the ONN in detail.

### 2.1. AE Model

The AE model [22] maps the input data to the hidden layer space to obtain its hidden layer representation, which can reconstruct the original input data through its hidden layer representations. AE is composed of an encoder *f*_**w**_1__(•) and a decoder *g*_**w**_2__(•), which can be expressed as

(1) $$\begin{array}{c} z=f_{w_{1}}\left(x\right), \end{array}$$

(2) $$\begin{array}{c} x{}^{\prime }=g_{w_{2}}\left(z\right). \end{array}$$

In the above equations, **x** and **x**′ are the input and reconstructed input, respectively; **z** and **x** are the hidden layer representations; and **w**_1_ and **w**_2_ are the parameters of the neural network, which can be obtained by minimizing the reconstruction error between **x** and **x**′ as follows:

(3) $$\begin{array}{c} \underset{w_{1},w_{2}}{\min}{\left\|x-x{}^{\prime }\right\|}_{2}^{2}. \end{array}$$

The hidden layer representation from AE is often used as an effective feature and directly input into the subsequent pattern recognition model.

### 2.2. SVM

One-class SVM is a widely used unsupervised anomaly detection method. It is actually a special form of SVM, which can learn a hyperplane to separate all data points in the kernel Hilbert space from the original one. Also, it maximizes the distance from the hyperplane to the original one. In the one-class SVM model, all data points except the original one are marked as positive samples, and the original ones are marked as negative samples. The training samples without labels are denoted as **X**, and the kernel Hilbert sparse is denoted as Φ(**X**). A hyperplane in the feature space is denoted as *f*(**X**_*n*:_)=*ω*^*T*^Φ(**X**_*n*:_) − *r*, which is used to separate from the original Φ(**X**_*n*:_),  *n* : 1,2,…, *N*, *ω* and *r* are normal vector and intercept of the hyperplane to be solved, respectively. In order to obtain the above two parameters, the following problem needs to be optimized:

(4) $$\begin{array}{c} \underset{w,r}{\min}\frac{1}{2}{\left\|w\right\|}_{2}^{2}+\frac{1}{v}\cdot \frac{1}{N}\sum_{n=1}^{N}\max\left(0,r-\langle w,\Phi \left(X_{n:}\right)\rangle \right)-r, \end{array}$$

where *v* ∈ (0,1) is the parameter used to weigh the importance of both the interval size and training error.

### 2.3. ONN Model

Based on one-class SVM, we now introduce the principle of ONN for unsupervised anomaly detection. This method can be regarded as a neural network structure designed using one-class SVM equivalent loss function. By constructing ONN, it is possible to utilize the features obtained from unsupervised transfer learning specifically used for anomaly detection. Then, it will be possible to identify anomalies in complex datasets where the positive and negative decision boundaries are highly nonlinear.

Specifically, this paper designs a simple feedforward CNN *F*(•), which has only one hidden layer and one output node. Afterwards, the objective function of ONN can be expressed as

(5) $$\begin{array}{c} \underset{w,r}{\min}\left[\frac{1}{2}{\left\|w\right\|}_{2}^{2}+\frac{1}{v}\cdot \frac{1}{N}\sum_{n=1}^{N}\max\left(0,r-\langle w,F\left(VX_{n:}\right)\rangle \right)+\frac{1}{2}{\left\|V\right\|}_{2}^{2}-r\right], \end{array}$$

where *w* represents the scalar output from the hidden layer to the output layer. Comparing equation (5) with equation (4), it can be found that 〈*w*, *F*(*V ***X**_*n*:_)〉 is used instead of 〈*w*, Φ(**X**_*n*:_)〉. Such change makes it possible to use the transfer learning function obtained by the AE and create an additional neural network layer to complete the function for anomaly detection. However, the cost of the change is that the objective function becomes nonconvex, so the model parameters cannot be globally optimized.

According to [23], it can be optimized by the alternate minimization method. First, the parameter *r* is fixed and *w*, *V* are optimized, and the following problem needs to be solved:

(6) $$\begin{array}{c} \underset{w,V}{\arg\min}\left[\frac{1}{2}{\left\|w\right\|}_{2}^{2}+\frac{1}{v}\cdot \frac{1}{N}\sum_{n=1}^{N}l\left(y_{n},{\overset{⌢}{y}}_{n}\left(w,V\right)\right)\;+\frac{1}{2}{\left\|V\right\|}_{2}^{2}\right], \end{array}$$

where $l\left(y,\overset{⌢}{y}\right)=\max\left(0,y-\overset{⌢}{y}\right)$, *y*_*n*_=*r*, ${\overset{⌢}{y}}_{n}\left(w,V\right)=\langle w,F\left(Vx_{n}\right)\rangle$. Similarly, the optimization can be expressed as

(7) $$\begin{array}{c} \underset{w,V}{\arg\min}\left[\frac{1}{Nv}\sum_{n=1}^{N}\max\left(0,r-{\overset{⌢}{y}}_{n}\right)\right]-r. \end{array}$$

In fact, for the parameters (*w*, *V*), the optimization can also use the standard backpropagation algorithm. The specific solution process can be found in [23]. Moreover, a convolutional self-encoding network can be used as a feature extractor to perform feature extraction on the original data and then input into the ONN. The convolutional self-encoding and ONN can be jointly optimized. After *r* is obtained, once the convergence is achieved, the decision function can be used to determine whether the sample is an abnormal one as follows:

(8) $$\begin{array}{c} S_{n}=\mathrm{sgn}\left({\overset{⌢}{y}}_{n}-r\right). \end{array}$$

### 2.4. Video Abnormal Event Detection Based on ONN

Inspired by the dual-stream neural network, the ONN model is trained separately on the local area blocks of the video frame and the optical flow graph to detect appearance anomalies and motion anomalies. Then, the two are merged to determine the final detection result.

Specifically, for the dense sampling of video frames, a deep AE is trained to obtain the input features, and the encoder layer of the pretrained autoencoder is copied and provided as input to the ONN. Then, the ONN parameters are jointly trained to obtain an appearance anomaly detection model. During the test, the densely sampled video frames are input into the model to get a normal appearance score ${\overset{⌢}{y}}_{\text{appearance}}$. In the same way, a motion detection model is trained for the corresponding optical flow image. The optical flow image corresponding to the video frame can be generated to obtain the motion anomaly ${\overset{⌢}{y}}_{\text{motion}}$. Then, we can score normally by appearance ${\overset{⌢}{y}}_{\text{appearance}}$ and abnormal movement score ${\overset{⌢}{y}}_{\text{motion}}$. A weight fusion and a preset threshold can be used to determine whether the area is abnormal:

(9) $$\begin{array}{c} S={\overset{⌢}{y}}_{\text{appearance}}+\alpha {\overset{⌢}{y}}_{\text{motion}}<\theta . \end{array}$$

## 3. Experiment and Discussion

This paper evaluates the performance of the proposed method on two video anomaly detection datasets published on the Internet, which are the USCD dataset [6] and the Subway dataset [7]. The USCD dataset provides frame-level annotations, so we use the area under the curve (AUC) of the receiver operating characteristic (ROC) curve measured according to the frame-level score as an evaluation indicator. For the Subway dataset, the frame-level annotations are not provided, and only event-level annotations are provided, so event-level evaluation criteria are used for evaluation on this dataset.

For the two datasets, each frame is adjusted to a size of 420 × 280, and the moving image is calculated by the optical flow method provided in [24]. In order to detect appearance anomalies and motion anomalies, RGB images and their corresponding video frame images are, respectively used, and two independent ONN networks are trained to detect appearance and motion anomalies. In the training phase, all images (including RGB images and dynamic flow graphs) are sampled through a sliding window with a size of 28 × 28 and a step length of 14. For each model, about 20000 image blocks are obtained as the final training set. In the test phase, the test samples are obtained through sliding windows of the same size and input into the model to calculate the results, which means that the final output size of each frame of image is 15 × 10 score map. In the AE, the encoder uses a common structure, while the decoder adopts the opposite structure. This means that 64-dimensional features are extracted from each 28 × 28 area and input into the hidden layer of ONN's 16 nodes. Then, the normal score is finally output. In the training phase, the batch size is set to 128, the initial learning rate is 0.001, and the training is up to 5000 iterations. Each layer initializes the weights [25] and uses ReLu as the activation function. The final fully connected layer is connected to a dropout layer. The whole method is implemented in Python and TensorFlow environment. The hardware conditions are as follows: NVIDIA GeForce GTX 1080Ti GPU, 32GB memory, and I7-9700 CPU.

### 3.1. Experimental Results on USCD Dataset

The UCSD anomaly dataset contains two subsets, PED1 and PED2, which were acquired from a static camera overlooking the sidewalk. An abnormal event is a nonpedestrian object (such as a vehicle) or an abnormal pedestrian movement. The main difference between the two subsets is the direction of the shooting angle of view (toward and away from the camera in PED1, and parallel to the camera plane in PED2). Some examples are shown in Figure 2. In addition, PED1 contains 34 normal and 36 abnormal videos with the sizes of 238 × 158, and each video clip contains 200 frames, while PED2 contains 12 normal and 16 abnormal videos with the sizes of320 × 240, and each video clip contains 150–200 frames.

In this dataset, the reference methods include Mixture of Dynamic Textures (MDT) [6], Sparse Reconstruction [8], Detection at 150FPS [1], and Appearance and Motion DeepNet (AMDN) [4]. The experimental results are shown in Table 1. Among them, the first two are manual features combined with anomaly detection models. AMDN [4] is a deep feature combined with anomaly detection models, and the last one is an end-to-end deep learning method. The results of the methods are obtained from their respective papers.

It can be seen from the results in Table 1 that the end-to-end deep learning method has the best detection performance, followed by the detection results of deep features + anomaly detection models. Also, the detection results of manual features + anomaly detection models are relatively poor. This is mainly because the two stages of feature extraction and model establishment in the end-to-end deep learning method are designed for the anomaly detection task, and the performance is improved after joint optimization. As an end-to-end deep learning method, the proposed method encapsulates the functions of feature extraction and ONN, so it has achieved good results. Specifically, the proposed method achieves 94.9% and 94.5% frame-level AUC on PED1 and PED2, which is better than all the reference methods.

It can be seen from Figure 3 that the proposed method can detect various types of abnormal events, including cycling on the sidewalk, the appearance of small cars and people walking on the lawn, etc.

### 3.2. Experiment Results on Subway Dataset

This dataset also contains two subsets, Entrance and Exit, which capture surveillance videos of the entrance door and exit door of the subway station, respectively. Their lengths are 96 minutes and 43 minutes, and each frame size is 512 × 384. The abnormal events in these two videos are mainly wrong directions (for example, passengers coming out of the entrance), failure to pay, loitering, unusual interactions (for example, one person walking awkwardly to avoid another person), and other situations (for example, sudden acceleration). Some samples from the dataset are shown in Figure 4. According to the annotation provided in [7], the training sample and the test sample are divided, that is, the first 15 minutes of the Entrance subset and the first 5 minutes of Exit subset are used as the training set, and the rest are used as the test set. It is worth noting that the experiments on the two subsets are performed independently.

Since this dataset does not provide frame-level annotation, this paper adopts the evaluation scheme in the literature [15] to determine the abnormal events in the experiment. In detail, a persistence algorithm is applied to the video sequence to locate local minima, where minima indicate an abnormal event. In order to reduce the possible impact of other events on the detection results, events near the occurrence time are combined into one abnormal event detection result. Reference methods used in this case include ground truth, dynamic sparse coding [26, 27] learning temporal regularity [3], and AMDN [4].

Table 2 shows the comparison of event-level detection results, which shows that our model has detected most abnormal events. Specifically, the proposed method detects at least one more event on the Entrance subset than other existing methods and has fewer false alarms. On the Exit subset, the proposed method and other methods detect all abnormal events, but only one false alarm is detected. The above results prove the effectiveness of the proposed method on the Subway dataset.  Figure 5 shows some correct detection results in this dataset.

## 4. Conclusion

In this paper, based on the idea of distance-based anomaly detection, we propose ONN-based method for video anomaly detection. Similar to one-class SVM, a type of neural network uses similar loss function training parameters, and its main advantage is that the features of the hidden layer are constructed for the specific task of anomaly detection. The proposed method is quite different from the recently proposed hybrid method that uses deep learning as a feature extractor and then separately trains anomaly detection models because the feature extraction in the hybrid method is general and not specific for anomaly detection tasks. Experimental results on two benchmark datasets show that the proposed method has both accuracy and robustness superiorities, confirming the its wide applicability in industrial and urban environments. The next research will consider using other information instead of optical flow diagram to represent the motion information of the videos.

## Figures and Tables

**Figure 1:** The procedure of video anomaly detection based on ONN.

**Figure 2:** Examples of normal events (a) and abnormal events (b) of UCSD dataset.

**Figure 3:** Examples of the detection results on the UCSD dataset.

**Figure 4:** Examples of normal events (a) and abnormal events (b) of Subway dataset.

**Figure 5:** Examples of the detection results on the Subway dataset.

**Table 1:** Comparison with the reference methods on the UCSD dataset.

Method	PED1	PED2
MDT	81.8	82.9
Sparse Reconstruction	87.6	86.3
Detection at 150FPS	91.8	—
AMDN	92.1	90.8
Proposed	**95.1**	**94.7**

**Table 2:** Comparison with the reference methods on the Subway dataset.

Method	Entrance		Exit	
	TP	FA	TP	FA
Ground truth	66	—	19	—
Dynamic sparse coding	60	4	19	2
Learning temporal regularity	61	5	17	5
AMDN	61	5	19	1
Proposed	62	3	19	1

## Data Availability

The datasets used in this paper can be accessed upon request.

## References

[1] Lu C., Shi J., Jia J. Abnormal event detection at 150 FPS in MATLAB.

[2] Sabokrou M., Fathy M., Hoseini M., Klette R. Real-time anomaly detection and localization in crowded scenes.

[3] Hasan M., Choi J., Neumanny J., Roy-Chowdhury A. K., Davis L. S. Learning temporal regularity in video sequences.

[4] Xu D., Yan Y., Ricci E., Sebe N. (2017). Detecting anomalous events in videos by learning deep representations of appearance and motion. *Computer Vision and Image Understanding*.

[5] Saligrama V., Chen Z. Video anomaly detection basedon local statistical aggregates.

[6] Mahadevan V., Li W., Bhalodia V., Vasconcelos N. Anomaly detection in crowded scenes.

[7] Adam A., Rivlin E., Shiimshoni I., Reinitz D. (2008). Robust real-time unusual event detection using multiple fixed location monitors. *IEEE Transactions on Pattern Analysis and Machine Intelligence*.

[8] Luo W., Liu W., Gao S. A revisit of sparse coding based anomaly detection in stacked RNN framework.

[9] Ren H., Liu W., Olsen S. I., Escalera S., Moeslund T. B. Unsupervised behavior-specific dictionary learning for abnormal event detection.

[10] Yiru Z., Bing D., Chen S., Liu Y., Lu H., Hua X.-S. Spatio-temporal autoencoder for video anomaly detection.

[11] Yuan Y., Fang J., Wang Q. (2015). Online anomaly detection in crowd scenes via structure analysis. *IEEE Transactions on Cybernetics*.

[12] Li W., Mahadevan V., Vasconcelos N. (2014). Anomaly detection and localization in crowded scenes. *IEEE Transactions on Pattern Analysis and Machine Intelligence*.

[13] Lecun Y., Bengio Y., Hinton G. (2015). Deep learning. *Nature*.

[14] Ravanbakhsh M., Nabi M., Mousavi H., Sangineto E., Sebe N. Plug-and-Play CNN for crowd motion analysis:an application in abnormal event detection.

[15] Ravanbakhsh M., Nabi M., Sangineto E., Marcenaro L., Regazzoni C., Sebe N. Abnormal event detection in videos using generative adversarial nets.

[16] Wang Y., Dai B., Hua G., Aston J., Wipf D. (2018). Recurrent variational autoencoders for learning nonlinear generative models in the presence of outliers. *IEEE Journal of Selected Topics in Signal Processing*.

[17] Zhao T., Li F., Tian P. (2020). A deep-learning method for device activity detection in mMTC under imperfect CSI based on variational-autoencoder. *IEEE Transactions on Vehicular Technology*.

[18] Kingma D. P., Welling M. Auto-encoding variational Bayes.

[19] Vincent P., Larcochele H., Bengio Y., Manzagol P.-A. Extracting and composing robust features with denoising autoencoders.

[20] Mei S., Montanari A., Nguyen P.-M. (2018). A mean field view of the landscape of two-layer neural networks. *Proceedings of the National Academy of Sciences*.

[21] Wang T., Snoussi H. (2014). Detection of abnormal visual events via global optical flow orientation histogram. *IEEE Transactions on Information Forensics and Security*.

[22] Sun C., Ma M., Zhao Z., Tian S., Yan R., Chen X. (2019). Deep transfer learning based on sparse autoencoder for remaining useful life prediction of tool in manufacturing. *IEEE Transactions on Industrial Informatics*.

[23] Chalathy R., Menon A. K., Chawla S. Anomaly detection using one-class neural networks.

[24] Baker S., Scharstein D., Lewis J. P., Roth S., Black M. J., Szeliski R. (2011). A database and evaluation methodology for optical flow. *International Journal of Computer Vision*.

[25] Glorot X., Bengio Y. Understanding the difficulty of training deep feedforward neural networks.

[26] Zhao B., Li F., Xing E. Online detection of unusual events in videos via dynamic sparse coding.

[27] Mehran R., Oyama A., Shah M. Abnormal crowd behavior detection using social force model.

